This article has been retracted.

# Effects of Transcranial Magnetic Stimulation Combined with Computer-Aided Cognitive Training on Cognitive Function of Children with Cerebral Palsy and Dysgnosia

**DOI:** 10.1155/2022/5316992

**Published:** 2022-08-26

**Authors:** Jun Chen, Xiaoming Yu, Guangjin Luo

**Affiliations:** Department of Rehabilitation, Qingdao Women and Children's Hospital, Qingdao, Shandong 266034, China

## Abstract

**Objective:**

This study is aimed at researching transcranial magnetic stimulation (TMS) effects combined with computer-aided cognitive training (CACT) on cognitive function of children suffering from cerebral palsy and dysgnosia.

**Methods:**

From December 2019 to October 2021, 86 children with cerebral palsy and dysgnosia who were treated at our hospital were recruited and assigned into observation and control groups (*n* = 43, each) using the random number table technique. The observation group received TMS combined with CACT (TMS+CACT), whereas the control group received only TMS. Chinese Wechsler Young Children Scale of Intelligence (C-WYCSI) and Chinese-Wechsler Intelligence Scale for Children (C-WISC) were used to evaluate the intelligence level of the two groups; Gross Motor Function Measure-88 (GMFM-88) of Fudan Chinese version was employed for evaluating the gross motor function of the two groups; a comparison was drawn among the two groups for the cerebral hemodynamic parameters before and after the treatment.

**Results:**

For young children, the verbal intelligence quotient (VIQ) scores at 6 and 12 weeks of treatment in the observation group were increased when compared to those in the control group (48.91 ± 3.70 vs. 47.32 ± 3.33, 54.25 ± 4.46 vs. 49.48 ± 3.36), and the observation group's performance intelligence quotient (PIQ) score at 12 weeks of treatment was higher as to that of the control group (65.38 ± 4.23 vs. 62.81 ± 4.74, all *P* < 0.05). For older age children, the observation group's VIQ and PIQ scores were greater than the control group's at 6 and 12 weeks of treatment, with statistical significance (63.80 ± 3.76 vs. 59.50 ± 5.32, 74.64 ± 12.04 vs. 65.08 ± 6.30; 63.91 ± 5.96 vs. 58.42 ± 3.70, 72.73 ± 5.06 vs. 66.42 ± 5.93; all *P* < 0.05). The GMFM-88 scale scores in both groups were increased after 6 and 12 weeks of treatment. After treatment for 12 weeks, the observation group's A-E scores were greater than those of the control group (all *P* < 0.05). The peak systolic velocity (*V*_s_), end-diastolic velocity (*V*_d_), and mean velocity (*V*_m_) at the anterior cerebral artery (ACA), middle cerebral artery (MCA), and posterior cerebral artery (PCA) in the observation group were dramatically increased than those in the control group (all *P* < 0.05) after 12 weeks of treatment.

**Conclusion:**

TMS+CACT can effectively improve the intelligence level, cognitive ability, gross motor function, and cerebral blood flow of children suffering from cerebral palsy and intellectual disability.

## 1. Introduction

Cerebral palsy is a common pediatric nervous system disorder that can lead to disability and deformity. Dysgnosia is a common complication of cerebral palsy. According to relevant research, the incidence of cerebral palsy complicated with dysgnosia is as high as 55%~65%. The more serious the condition of children is, the more likely they are to be complicated with dysgnosia. Children with cerebral palsy and dysgnosia often show motor dysfunction, intellectual developmental disorder, and cognitive dysfunction, which can seriously affect their physical health and quality of life [1, 2]. Currently, no effective method for treating cerebral palsy exists. The key to the treatment of cerebral palsy with dysgnosia is to improve the level of children's intelligence, motor, and cognitive function. Routine rehabilitation intervention is often adopted in the clinical treatment of cerebral palsy with dysgnosia, but the treatment effect is not evident. Repetitive transcranial magnetic stimulation (rTMS) is a novel type of neuroelectrophysiological technology, which is painless, noninvasive, easy to operate, and very safe. It can generate a certain intensity of time-varying magnetic field in a specific part outside the skull, induce an electric field in the brain, cause induced current, stimulate the nearby nerve tissue, and further affect the brain metabolism and the physiological hormone of neuroelectric activity. Currently, this technology has been widely used in the fields of psychological diseases and nervous system diseases [3, 4]. Cognitive training is a method that specialized doctors are responsible for or using computer platform to complete training items, including attention training, memory training, processing speed training, and flexibility training. It is easy to operate and has good compliance. Computer-aided cognitive training (CACT) is more convenient for children to train at home [5, 6]. The objective of this research was to explore the effects of TMS+CACT on cognitive function of children suffering from cerebral palsy and dysgnosia. The following is the report.

## 2. Materials and Methods

### 2.1. General Data

From December 2019 to October 2021, 86 children with cerebral palsy complicated by dysgnosia were treated in our hospital as outpatients or inpatients and were registered and randomized into observation and control groups utilizing the random number table method, having 43 cases in every group. The observation group had 25 males and 18 females; their ages ranged from 3 years and 11 months to 7 years, with an average of 67.07 ± 7.89 months; dysgnosia grade: mild in 17 cases, moderate in 20 cases, and severe in 6 cases; clinic classification of cerebral palsy: 33 cases of spastic type, 7 cases of mixed type, 2 cases of dyskinetic type, and 1 case of ataxic type. There were 22 males and 21 females in the control group; with an average of 68.30 ± 12.76 months, their ages were from 3 years and 11 months to 8 years; dysgnosia grade: mild in 18 cases, moderate in 18 cases, and severe in 7 cases; clinic classification of cerebral palsy: 30 cases of spastic type, 9 cases of mixed type, 3 cases of dyskinetic type, and 1 case of ataxic type. The general data of the two groups were comparable (all *P* > 0.05). The Hospital Ethics Committee gave its approval to this study. Diagnostic criteria: the diagnostic criteria and clinic classification of cerebral palsy were in line with the standards formulated by the Compilation Committee of *Guidelines for Rehabilitation and Treatment of Cerebral Palsy in China* [7] and conform to the classification guidelines for cerebral palsy in the *World Health Organization International Classification of Functioning*, *Disability*, *and Health* [8]. The diagnosis of dysgnosia conformed to the diagnostic criteria of intellectual developmental disorder in the *International Classification of Diseases 11th Revision (ICD-11)* [9]. Inclusion criteria: (1) all met the Western and Chinese diagnostic criteria; (2) age ≥ 3 years and 11 months; (3) the child was conscious and his/her vital signs were stable; (4) the study was voluntarily undertaken by all of the enrolled children and their families. Exclusion criteria: (1) children with central brain injury caused by progressive diseases such as cerebral edema and viral encephalitis; (2) children with water and electrolyte disorders; (3) children with epilepsy; (4) children with severe lung infection; (5) children with systemic immune system diseases; and (6) children suffering from extreme organ diseases such as heart, liver, and kidney dysfunctions.

### 2.2. Therapies

Both groups received routine rehabilitation training. The TMS+CACT was administered to the observation group, and the control group got administered by TMS only. TMS: the children were treated with TMS instrument with positioning treatment cap. The stimulation frequency was adjusted to 5-10 Hz, the stimulation intensity was 80%-100% resting state motion threshold (RMT), and the stimulation sites were F3 and F4 of EEG 10-20 system. The treatment was given once daily for 20 minutes, 5 times a week, and 20 times as a course. The treatment lasted for 3 courses. CACT: computer interactive table rehabilitation cognitive training software and MindWave Mobile Core attention training software were used to train the children's memory, executive, attention, and spatial vision abilities. The training content included (1) attention training: selecting the picture that was consistent with the reference picture from the screen pictures and selecting the picture from simple to complex; (2) memory training: including graphic memory and detail memory, memorizing screen pictures or texts, and answering relevant questions; (3) time and place orientation training: children are trained according to instructions or scene graphics; and (4) visual space and executive function training: in different content and different number of picture groups, selecting rotated reference pictures as visual space function training, and stick figure drawing as executive function training. In accordance with the type and severity of cognitive impairment, different combinations were used to conduct cognitive function training for patients; the training was provided once daily for 30 minutes, 5 times a week, while the training lasted for 12 weeks.

### 2.3. Observational Indexes

(1) Intelligence level: before and after treatment, the intelligence level of the younger children (3 years and 11 months to 6 years old) was evaluated by the Chinese Wechsler Young Children Scale of Intelligence (C-WYCSI) [10], while that of older children (6 to 16 years old) was assessed by Chinese-Wechsler Intelligence Scale for Children (C-WISC) [11]. Both sets of intelligence assessment tools had high reliability and validity. Each set of intelligence scale included two parts: speech and operation, and consists of 11 subitems, such as picture vocabulary, arithmetic, picture generalization, comprehension, animal laying eggs, picture filling, maze, visual analysis, wood block pattern, and geometric figure. The results of intelligence assessment include verbal intelligence quotient (VIQ) and performance intelligence quotient (PIQ), which are completed by professional testers in the Neurorehabilitation Department of the hospital. (2) Gross motor ability: before and after treatment, the gross motor function was evaluated by GMFM-88 Scale of Fudan Chinese version [12]. The scale had 88 items, which were distributed in 5 functional areas: (A) lying motion and turning over (17 items); (B) sitting motion (20 items); (C) crawling and kneeling motion (14 items); (D) standing (13 items); and (E) walking, running, and jumping (24 items). The score of each item was 0~3 points according to the degree of completion, and score for each functional area was obtained. The greater the child's gross motor performance, the higher the score. In order to reduce the error, the same doctor conducted blind evaluation before and after the treatment. (3) Comparison of the two groups' cerebral hemodynamic parameters before and after the treatment: color Doppler ultrasound was employed to evaluate peak systolic velocity (*V*_s_), end-diastolic velocity (*V*_d_), and mean velocity (*V*_m_) at the anterior cerebral artery (ACA), middle cerebral artery (MCA), and posterior cerebral artery (PCA) before and after treatment in both groups.

### 2.4. Statistical Methods

The data were analyzed and processed using SPSS 20.0 statistical software. ^−^*x* ± *s* was used to represent the measurement data. The intergroup comparison was executed with an independent sample *t*-test, while the intragroup comparison was done with a paired *t*-test before and after treatment. The *χ*^2^ test was performed on the counting data, which was expressed as frequency and constituent ratio. A statistically significant difference was represented by *P* < 0.05.

## 3. Results

### 3.1. Comparison of C-WYCSI Scores of Young Children between Two Groups before and after Treatment

The VIQ and PIQ scores did not vary significantly among the two groups before treatment (both *P* > 0.05); however, VIQ and PIQ scores were higher in both groups after being treated for 3, 6, and 12 weeks. At 6 and 12 weeks of treatment, the observation group's VIQ score was greater than that of the control group, and the observation group's PIQ score was higher compared to the control group's at 12 weeks of treatment, both with statistical significance (all *P* < 0.05, Table 1).

### 3.2. Comparison of C-WISC Scores of the Older Children between Two Groups before and after Treatment

The VIQ and PIQ scores did not change significantly among the two groups prior to treatment (both *P* > 0.05). However, at 3, 6, and 12 weeks of treatment, the scores for VIQ and PIQ in the observation group and PIQ in the control group increased. After receiving treatment for 6 and 12 weeks, the control group's VIQ score improved. At 6 and 12 weeks after treatment, the observation group's VIQ and PIQ scores were greater than those of the control group, with statistical significances (all *P* < 0.05, Table 2).

### 3.3. Comparison of GMFM-88 Scale Scores between Two Groups before and after Treatment

The exercise ability scores among the two groups prior to treatment did not differ significantly (*P* > 0.05). Exercise ability scores, however, in both groups improved after receiving treatment for 6 and 12 weeks. The observation group's A~E scores were substantially greater than those of the control group following treatment for 12 weeks (all *P* < 0.05, Table 3).

### 3.4. Comparison of Cerebral Hemodynamic Parameters between Two Groups before and after Treatment

Prior to the treatment, no major differences could be observed among the two groups in the *V*_s_, *V*_d_, and *V*_m_ parameters of the ACA, MCA, and PCA (all *P* >0.05). *V*_s_, *V*_d_, and *V*_m_ of ACA, MCA, and PCA in both the groups, however, improved after treatment for 6 and 12 weeks. *V*_s_, *V*_d_, and *V*_m_ of ACA, MCA, and PCA in the observation group were considerably greater compared to those in the control group after receiving treatment for 12 weeks (all *P* < 0.05, Table 4).

## 4. Discussion

Cerebral palsy is a refractory disease with a long course. Children with cerebral palsy often have perceptual, behavioral, sensory, cognitive, and other disorders, as well as varying degrees of mental retardation. If not treated in time, it may lead to lifelong disability and bring heavy burden to the family and society. The clinical treatment of cerebral palsy mostly adopts comprehensive treatment methods including physical therapy and cognitive function training. The working principle of TMS is to send pulse electric current into the coil and then generate pulse magnetic field around the coil. The induced current in the head is generated by the pulse magnetic field, which then activates the associated brain nerve units [13, 14]. The effects of different TMS frequencies on cortical metabolism and cerebral blood flow may vary. High-frequency stimulation can improve cerebral perfusion and local cerebral blood flow and metabolism, while low-frequency stimulation can reduce cerebral blood flow and metabolism. Compared with conventional electrical stimulation, TMS has the following characteristics: (1) easy to achieve deep brain stimulation. Surface electrode stimulation can make the electric field diffused rapidly and could not reach the deep brain. Implanting electrical stimulation cannot be extensively employed in clinical practice because it is traumatic, and the loss of magnetism in bone and muscle is small, due to which TMS can reach deep into the brain. (2) Less discomfort: electrical stimulation has strong stimulation to scalp and skull and can make the person produces strong discomfort. TMS does not act directly on nerves but can stimulate them by producing induced electrical current. The size of the induced current is inversely proportional to the resistance. There is no discomfort when induced current is applied to bone and scalp with large resistance. (3) Not direct contact with human body: magnetic stimulation equipment does not make direct contact with the human body, which can reduce the risk of injury to the human body. CACT began to appear in the 1990s and has been extensively utilized for treating cerebral infarction, brain injury, and other neurological diseases currently. Compared with traditional manual training, CACT has the following advantages. (1) By combining cognitive training with fun animations, it makes the treatment process more interesting through visual, auditory, tactile, and other multimedia technologies, which can better attract the attention and improve the cognitive function of children. (2) Through the standardized intervention method of the programmed training task module, it has strong repeatability and is easy to compare and promote the efficacy. (3) Individualized treatment plans can be developed according to the specific conditions of children. Real-time data analysis feedback can also be carried out in the training process, which can effectively stimulate the training enthusiasm of children and is conducive to follow-up rehabilitation.

TMS combined with CACT was utilized for treating the observation group in the present study. The observation group's VIQ score was greater than the control group's at 6 and 12 weeks, and the observation group's PIQ score was higher than that of the control group at 12 weeks, according to the results. At 6 and 12 weeks following treatment, the older children in the observation group had superior VIQ and PIQ scores than the control group. The observation group's scores of the A~E item on the GMFM-88 scale were greater than the control group's after 12 weeks of treatment, showing that TMS+CACT can successfully enhance the intelligence level and motor function of children suffering from cerebral palsy complicated by dysgnosia. Intracranial blood flow in children with brain injury is characterized by low speed and high resistance, showing sustained hypoperfusion and low circulation, which can affect the continued brain development of infants and young children. TMS can effectively improve the brain tissue perfusion in children with brain injury and promote their neuropsychological development [15]. According to relevant studies, TMS can effectively improve the motor function of children suffering from cerebral palsy. In other studies, TMS was applied to children with dysgnosia and showed significant effects [16]. Cognitive training can enhance synaptic efficiency and promote neural function reorganization, and children can improve their cognitive ability through repetitive exercises [17]. In the present study, the combined application of TMS and CACT further improved the children's intelligence, motor ability, and cognitive ability. TMS+CACT can effectively expand the cerebral vascular microcirculation, stimulate the activity of neurons and cells in the brain, and improve the intelligence and motor ability of children. TMS+CACT can effectively regulate the levels of serum markers related to cerebral nerve function in children. The stimulation coil of TMS instrument can generate the corresponding magnetic field, and the magnetic field through the skull will generate the corresponding induction current and finally play the role of regulating local neurons, which further promotes the recovery of brain nerve.

Dysgnosia in children with cerebral palsy is mostly caused by brain injury. Abnormal cerebral blood flow parameters can reflect the severity of brain injury and affect intellectual development [18, 19]. According to relevant studies, children with cerebral palsy with cerebral microcirculation disorders have slow cerebral artery blood flow and increased vascular resistance, which further influences dysgnosia [20]. Cerebral blood flow velocity is closely related to changes in local cerebral blood flow. Peak flow velocity and average flow velocity can be regarded as relative indicators of cerebral blood flow, and average flow velocity can reflect the degree of cerebrovascular filling. At 6 and 12 weeks of treatment, *V*_s_, *V*_d_, and *V*_m_ of ACA, MCA, and PCA improved in both groups. *V*_s_, *V*_d_, and *V*_m_ of ACA, MCA, and PCA in the observation group were considerably greater compared to those in the control group after treatment for 12 weeks (all *P* < 0.05). This indicates that repeated TMS combined with CACT can effectively improve cerebral blood flow, cerebral blood flow microcirculation disorder, and brain injury, repair the blood-brain barrier, and improve the intellectual development of children with cerebral palsy combined with dysgnosia. Multiple previous studies have shown that repetitive transcranial stimulation has an impact on cortical metabolism and cerebral blood flow in children suffering from cerebral palsy [21, 22]. This is supported by the findings of the current investigation. In the observation group, repeated TMS plus CACT was used and further improved the cerebral blood flow.

In conclusion, TMS+CACT has a good therapeutic effect and clinical application value in children with cerebral palsy complicated by dysgnosia, improving motor functions, intelligence levels, and cerebral blood flow.

## Figures and Tables

**Table 1:** Comparison of C-WYCSI scores of young children between two groups before and after treatment (^−^*x* ± *s*, points).

Group	VIQ score				PIQ score			
	Before treatment	Treatment for 3 weeks	Treatment for 6 weeks	Treatment for 12 weeks	Before treatment	Treatment for 3 weeks	Treatment for 6 weeks	Treatment for 12 weeks
Observation group (*n* = 32)	42.69 ± 3.65	46.09 ± 3.28^a^	48.91 ± 3.70^a^	54.25 ± 4.46^a^	52.84 ± 4.64	57.16 ± 4.86^a^	60.78 ± 4.18^a^	65.38 ± 4.23^a^
Control group (*n* = 31)	41.71 ± 3.51	44.81 ± 3.35^a^	47.32 ± 3.33^a^	49.48 ± 3.36^a^	52.13 ± 4.11	57.16 ± 3.48^a^	59.52 ± 3.33^a^	62.81 ± 4.74^a^
*t* value	1.083	1.542	1.783	4.778	0.646	0.005	1.327	2.269
*P* value	0.283	0.128	0.080	<0.001	0.521	0.996	0.190	0.027

Note: compared with before treatment, ^a^*P* < 0.05.

**Table 2:** Comparison of C-WISC scores of the older children between two groups before and after treatment (^−^*x* ± *s*, points).

Group	VIQ score				PIQ score			
	Before treatment	Treatment for 3 weeks	Treatment for 6 weeks	Treatment for 12 weeks	Before treatment	Treatment for 3 weeks	Treatment for 6 weeks	Treatment for 12 weeks
Observation group (*n* = 11)	51.55 ± 2.66	57.55 ± 4.08^a^	63.82 ± 3.76^a^	74.64 ± 12.04^a^	53.82 ± 4.53	60.55 ± 4.78^a^	63.91 ± 5.96^a^	72.73 ± 5.06^a^
Control group (*n* = 12)	50.92 ± 6.76	55.33 ± 5.87	59.50 ± 5.32^a^	65.08 ± 6.30^a^	53.25 ± 2.86	56.58 ± 3.34^a^	58.42 ± 3.70^a^	66.42 ± 5.93^a^
*t* value	0.298	1.040	2.228	2.414	0.363	2.320	2.681	2.732
*P* value	0.770	0.310	0.037	0.025	0.721	0.031	0.014	0.012

Note: compared with before treatment, ^a^*P* < 0.05.

**Table 3:** GMFM-88 scores before and after treatment (^−^*x* ± *s*, points).

Group	A				B				C				D				E			
	Before treatment	Treatment for 3 weeks	Treatment for 6 weeks	Treatment for 12 weeks	Before treatment	Treatment for 3 weeks	Treatment for 6 weeks	Treatment for 12 weeks	Before treatment	Treatment for 3 weeks	Treatment for 6 weeks	Treatment for 12 weeks	Before treatment	Treatment for 3 weeks	Treatment for 6 weeks	Treatment for 12 weeks	Before treatment	Treatment for 3 weeks	Treatment for 6 weeks	Treatment for 12 weeks
Observation group (*n* = 34)	32.84 ± 3.29	36.37 ± 2.84^a^	41.55 ± 2.65^a^	50.12 ± 4.60^a^	16.84 ± 1.09	22.47 ± 2.51^**a**^	28.49 ± 2.55^**a**^	35.30 ± 3.20^a^	6.53 ± 2.26	9.49 ± 2.11^**a**^	13.51 ± 2.32^**a**^	17.21 ± 1.58^a^	5.00 ± 1.29	8.28 ± 2.25^**a**^	11.44 ± 2.46^**a**^	16.65 ± 3.65^a^	2.74 ± 0.95	4.63 ± 1.23^**a**^	6.51 ± 1.47^**a**^	9.23 ± 2.38^a^
Control group (*n* = 43)	32.56 ± 2.93	37.21 ± 2.53^a^	40.81 ± 2.75^a^	44.23 ± 2.83^a^	16.51 ± 1.20	19.98 ± 2.27^**a**^	25.00 ± 2.80^**a**^	30.74 ± 4.21^a^	6.30 ± 1.39	6.88 ± 1.33	9.37 ± 1.80^a^	13.28 ± 4.28^a^	5.21 ± 1.30	6.95 ± 1.09^**a**^	8.14 ± 1.34^**a**^	10.95 ± 2.48^a^	2.65 ± 0.92	3.65 ± 0.92^**a**^	4.53 ± 1.16^**a**^	6.60 ± 1.76^a^
*t* value	0.415	1.444	1.277	7.141	1.316	4.818	6.038	5.650	0.575	6.849	9.236	5.644	0.749	3.477	7.728	8.468	0.460	4.155	6.918	5.822
*P* value	0.679	0.152	0.205	<0.001	0.192	<0.001	<0.001	<0.001	0.567	<0.001	<0.001	<0.001	0.456	0.001	<0.001	<0.001	0.647	<0.001	<0.001	<0.001

Note: compared with before treatment, ^a^*P* < 0.05. A: lying motion and turning over; B: sitting motion; C: crawling and kneeling motion; D: standing; E: walking, running, and jumping.

**Table 4:** Comparison of cerebral hemodynamic parameters between two groups before and after treatment (^−^*x* ± *s*).

Group	ACA				MCA				PCA			
	Before treatment	Treatment for 3 weeks	Treatment for 6 weeks	Treatment for 12 weeks	Before treatment	Treatment for 3 weeks	Treatment for 6 weeks	Treatment for 12 weeks	Before treatment	Treatment for 3 weeks	Treatment for 6 weeks	Treatment for 12 weeks
*V*_s_												
Observation group (*n* = 34)	60.20 ± 8.34	67.33 ± 5.23^**a**^	74.59 ± 5.40^**a**^	82.90 ± 7.93^**a**^	69.23 ± 6.98	76.55 ± 5.28^**a**^	82.38 ± 4.90^**a**^	89.75 ± 7.20^**a**^	52.31 ± 4.39	56.87 ± 4.43^**a**^	60.47 ± 4.43^**a**^	66.63 ± 4.79^**a**^
Control group (*n* = 43)	58.39 ± 5.81	64.60 ± 5.18^**a**^	69.69 ± 5.18^**a**^	76.65 ± 7.55^**a**^	68.14 ± 4.74	74.06 ± 4.69^**a**^	79.44 ± 4.42^**a**^	84.29 ± 5.23^**a**^	51.23 ± 4.02	55.56 ± 3.11^**a**^	59.54 ± 3.16^**a**^	64.59 ± 3.94^**a**^
*t* value	1.168	2.437	4.295	3.741	0.852	2.319	2.924	4.026	1.189	1.584	1.117	2.156
*P* value	0.247	0.017	<0.001	<0.001	0.397	0.023	0.004	<0.001	0.238	0.117	0.267	0.034
*V*_d_												
Observation group (*n* = 34)	21.43 ± 5.46	28.10 ± 3.96^**a**^	32.05 ± 3.88^**a**^	38.32 ± 5.30^**a**^	24.36 ± 5.40	30.57 ± 2.55^**a**^	33.57 ± 2.83^**a**^	38.09 ± 3.36^**a**^	15.21 ± 4.70	19.61 ± 4.40^**a**^	23.61 ± 4.26^**a**^	30.39 ± 6.83^**a**^
Control group (*n* = 43)	22.41 ± 3.41	26.69 ± 2.30**a**	29.58 ± 3.03^**a**^	33.62 ± 4.42^**a**^	23.67 ± 3.83	25.46 ± 3.90^**a**^	30.30 ± 3.77^**a**^	34.63 ± 4.88^**a**^	14.11 ± 2.82	17.46 ± 2.75^**a**^	20.80 ± 2.54^**a**^	24.23 ± 3.42^**a**^
*t* value	1.003	2.017	3.300	4.475	0.688	7.191	4.553	3.824	1.315	2.717	3.719	5.287
*P* value	0.319	0.048	0.001	<0.001	0.493	<0.001	<0.001	<0.001	0.193	0.008	<0.001	<0.001
*V*_m_												
Observation group (*n* = 34)	35.36 ± 3.41	39.81 ± 2.30^**a**^	43.52 ± 3.72^**a**^	49.27 ± 3.75^**a**^	41.88 ± 4.51	47.84 ± 3.03^**a**^	51.76 ± 3.49^**a**^	57.17 ± 4.67^**a**^	26.78 ± 1.79	28.76 ± 1.75^**a**^	33.20 ± 5.01^**a**^	36.51 ± 5.78^**a**^
Control group (*n* = 43)	36.01 ± 4.42	40.27 ± 2.80^**a**^	43.08 ± 2.19^**a**^	46.42 ± 3.32^**a**^	41.02 ± 3.29	41.87 ± 3.19	46.77 ± 2.76^**a**^	49.79 ± 2.89^**a**^	26.11 ± 1.94	28.34 ± 1.19^**a**^	29.99 ± 1.74^**a**^	32.37 ± 2.30^**a**^
*t* value	0.770	0.837	0.673	3.721	1.008	8.914	7.353	8.811	1.672	1.282	3.971	4.364
*P* value	0.443	0.405	0.503	<0.001	0.316	<0.001	<0.001	<0.001	0.098	0.203	<0.001	<0.001

Note: compared with before treatment, ^a^*P* < 0.05.

## Data Availability

The labeled dataset used to support the findings of this study is available from the corresponding author upon request.

## References

[1] Wimalasundera N., Stevenson V. L. (2016). Cerebral palsy. *Practical Neurology*.

[2] Gulati S., Sondhi V. (2018). Cerebral palsy: an overview. *Indian Journal of Pediatrics*.

[3] Lefaucheur J. P., Aleman A., Baeken C. (2020). Evidence-based guidelines on the therapeutic use of repetitive transcranial magnetic stimulation (rTMS):An update (2014-2018). *Clinical Neurophysiology*.

[4] Aloizou A. M., Pateraki G., Anargyros K. (2021). Transcranial magnetic stimulation (TMS) and repetitive TMS in multiple sclerosis. *Reviews in the Neurosciences*.

[5] Youze H., Ting Y., Yaqi B., Tianshen X., Tiecheng W., Jingsong W. (2021). Computer aided self-regulation learning and cognitive training improve generalization ability of patients with poststroke cognitive impairment. *Scientific Reports*.

[6] Otsuka T., Tanemura R., Noda K., Nagao T., Sakai H., Luo Z. W. (2015). Development of Computer-aidedcognitive training program for elderly and its effectivenessthrougha 6 months group intervention study. *Current Alzheimer Research*.

[7] Li X., Tang J., Ma B., Qin J., Zou L., Wang J. (2014). Definition, diagnostic criteria and clinical classification of cerebral palsy. *Chinese Journal of Practical Pediatrics*.

[8] Rosenbaum P., Stewart D. (2004). The World Health Organization international classification of functioning, disability, and health: a model to guide clinical thinking, practice and research in the field of cerebral palsy. *Seminars in Pediatric Neurology*.

[9] Oltmanns J. R. (2021). Personality traits in the international classification of diseases 11th revision (ICD-11). *Current Opinion in Psychiatry*.

[10] Yaoxian G., Xiaoyang D. (1986). *Chinese Webster’s Intelligence Scale Guidance Manual for Young Children*.

[11] Yaoxian G., Taisheng C. (1996). *China Wechsler Intelligence Scale for Children (C-WISC) Instruction Manual*.

[12] Wei S. (2018). Study on item difficulty improvement and responsiveness and precision of the Chinese version of the Fudan gross motor function test scale for cerebral palsy. *Chinese Journal of Evidence-Based Pediatrics*.

[13] Hameed M. Q., Dhamne S. C., Gersner R. (2017). Transcranial magnetic and direct current stimulation in children. *Current Neurology and Neuroscience Reports*.

[14] Krajnc N., Zidar J. (2016). The role of transcranial magnetic stimulation in evaluation of motor cortex excitability in Rett syndrome. *European Journal of Paediatric Neurology*.

[15] Inoue Y. (2016). Repetitive transcranial magnetic stimulation (rTMS) for higher brain function deficits. *Brain and Nerve*.

[16] Lihua M., Ying C., Xing Y. (2021). Effects of repetitive transcranial magnetic stimulation combined with sandplay therapy on intelligence improvement and cognitive development in mentally retarded children. *Journal of Clinical and Experimental Medicine*.

[17] Bao J. S., Tong G. L., Zhou T. C., Yi X. (2018). Study on the effect of Tiaoshen Tongdu acupuncture combined with cognitive function training on children with cerebral palsy. *Sichuan Traditional Chinese Medicine*.

[18] Gorbachev V. I., Bragina N. V., Gorbachev S. V. (2019). About interrelation of intracranial pressure and cerebral blood flow when positioning at patients with acute brain damage. *Regional Blood Circulation and Microcirculation*.

[19] Cammarota G., Verdina F., Lauro G. (2021). Neurally adjusted ventilatory assist preserves cerebral blood flow velocity in patients recovering from acute brain injury. *Journal of Clinical Monitoring and Computing*.

[20] Niu N., Tang Y., Hao X., Wang J. (2020). Non-invasive evaluation of brain death caused by traumatic brain injury by ultrasound imaging. *Frontiers in Neuroinformatics*.

[21] Turner D. A., Degan S., Galeffi F., Schmidt S., Peterchev A. V. (2021). Rapid, dose-dependent enhancement of cerebral blood flow by transcranial AC stimulation in mouse. *Brain Stimulation*.

[22] Hoover E. M., Crouzet C., Bordas J. M. (2021). Transcranial chronic optical access to longitudinally measure cerebral blood flow. *Journal of Neuroscience Methods*.

